The article "Down-regulation of XIAP enhances the radiosensitivity of esophageal cancer cells in vivo and in vitro" was retracted in 2021. Reasons: fabricated or falsified data; manipulated images; an official misconduct investigation; misconduct by an author.

# Down-regulation of XIAP enhances the radiosensitivity of esophageal cancer cells *in vivo* and *in vitro*

**DOI:** 10.1042/BSR20170711

**Published:** 2017-09-19

**Authors:** Xin Wen, Xin-Rui Han, Shao-Hua Fan, Zi-Feng Zhang, Lu Chen, Gao Yi, Dong-Mei Wu, Jun Lu, Yuan-Lin Zheng

**Affiliations:** 1 Key Laboratory for Biotechnology on Medicinal Plants of Jiangsu Province, School of Life Science, Jiangsu Normal University, Xuzhou 221116, P.R. China; 2 Department of Oncology, Linyi Cancer Hospital, Linyi 276000, P.R. China

**Keywords:** Esophageal cancer, Gene silencing, Radiosensitivity, siRNA, Viability, XIAP

## Abstract

The study investigated the effects of X-chromosome-linked inhibitor of apoptosis (*XIAP*) gene silencing on the radiosensitivity of esophageal cancer (EC) cells. Western blotting was used to select EC cell lines with XIAP overexpression. Selected EC9706 and KYSE30 cell lines were both divided into four groups: the blank control group, the negative control (NC) group (transfected with pBSHH1), the siRNA-enhanced group (transfected with pBSHH1-XIAP1-siRNA), and the siRNA-decreased group (transfected with pBSHH1-XIAP2-siRNA). Expressions of XIAP were measured by reverse-transcription quantitative PCR (RT-qPCR) and Western blotting, cell survival and viability by MTT assay and colony formation assay, and cell apoptosis by flow cytometry, respectively. Caspase-3 and caspase-9 activity were detected using caspase-3 and caspase-9 activity detection kits. A nude mice model of EC9706 cell line was established to measure tumorigenesis ability. Compared with the NC group, *XIAP* mRNA and protein expressions were decreased, caspase-3 and caspase-9 activity and apoptosis were up-regulated, and cell survival rate and colony-forming efficiency were lower in the siRNA-enhanced and siRNA-decreased groups in both the cell lines; while the opposite trends were found in the siRNA-decreased group compared with the siRNA-enhanced group. Tumor weight and volume of nude mice were decreased in the siRNA-enhanced and siRNA-decreased groups than those in the NC group, and were elevated in the siRNA-decreased group compared with the siRNA-enhanced group. These results indicate that *XIAP* gene silencing would strengthen the radiosensitivity of EC9706 cells, which provides a novel target for the treatment of EC.

## Introduction

As one of the most frequent malignancies, esophageal cancer (EC) ranks amongst the top six the most dominating causes of cancer-related deaths worldwide [1]. Geographically, EC exhibits high incidences in some regions especially China like Taihang Mountain area in Henan, the southern area in Fujian (Minnan area), and Chaoshan plain in Guangdong Province as well [2]. Moreover, the incidence of EC grows with age, with lowest peak at the age of 30 and highest peak at the age of 60 [3]. In addition, various factors are linked to EC occurrence, including the consumption of alcohol and hot beverages, nutritional deficiency of some minerals and vitamins, opium smoking, various nitrosamine-containing foodstuffs as well as human papilloma virus (HPV) infection [3]. Generally, surgery is the main treatment for resectable EC, and for EC patients with lymph node (LN) metastasis, postoperative radiotherapy serves as an effective way to increase the survival rate and reduce the recurrence rate [4]. Unfortunately, even though surgery and radiotherapy were applied for EC patients, the 5-year survival rate is still poor [5]. Interestingly, several studies reported that some tumor-related genes mediating some RNAs are able to contribute to important effects on suppression or promotion of radiosensitivity in EC [6–8]. Thus, it is of great significance to find new therapeutic methods involving tumor-related genes to improve the prognosis in EC patients.

The article "Down-regulation of XIAP enhances the radiosensitivity of esophageal cancer cells in vivo and in vitro" was retracted in 2021. Reasons: fabricated or falsified data; manipulated images; an official misconduct investigation; misconduct by an author.

On behalf of the crucial regulator of apoptosis, inhibitor of apoptosis proteins (IAPs) function their ability via binding to caspases which mainly execute apoptosis, so as to inhibit their catalytic ability [9]. Particularly, X-chromosome-linked inhibitor of apoptosis (XIAP) is an indispensable member of the IAP family and has been proven to be an efficient endogenous caspase inhibitor amongst the IAPs [10]. In recent years, XIAP has participated in developing new cancer therapeutics, since XIAP is greatly expressed in different kinds of human cancers but not expressed or less expressed in normal tissues [11–13]. Besides, down-regulation or inhibition of XIAP through different ways has been successful in many tumors such as prostate cancer [14] and hepatocellular carcinoma [15]. Furthermore, suppression of XIAP expression via oligonucleotides or siRNA inhibits the proliferation and invasion of tumor cells, and enhances the apoptosis of tumor cells, thereby suppressing tumor growth [16]. According to previous studies, the transfection of siRNA targetting XIAP in tumor cells is closely correlated with the radiation sensitivity [17,18]. Gene silencing for tumor-suppressor genes is a vital event in the development of cancer and can be functioned by inhibiting mutation or by shutting down the promoter region and sites where gene transcription begins [19]. Therefore, we performed the performed study to investigate effects of *XIAP* gene silencing on the radiosensitivie EC cells.

## Materials and methods

### Ethics statement

The experimental procedures were conducted in accordance with the Ethics Committee for Experiments on Animals of Laboratory Animal Center of Key Laboratory for Biotechnology on Medicinal Plants of Jiangsu Province, School of Life Science, Jiangsu Normal University.

The article "Down-regulation of XIAP enhances the radiosensitivity of esophageal cancer cells in vivo and in vitro" was retracted in 2021. Reasons: fabricated or falsified data; manipulated images; an official misconduct investigation; misconduct by an author.

### Cell culture

Human EC cell lines EC9706, TE10, KYSE70, KYSE510, and KYSE30 were preserved in our laboratory. *Escherichia coli* strain JM109 was purchased from TAKARA Bio Inc. (Shiga, Japan). The pBSHH1 plasmid was purchased from Shanghai ZJ Bio-Tech Co., Ltd. (Shanghai, China). EC9706, TE10, KYSE70, KYSE510, and KYSE30 cells were conventionally cultured in a 5% CO_2_ incubator containing the Roswell Park Memorial Institute 1640 medium (RPMI 1640; Gibco BRL Co. Ltd, Gaithersburg, Maryland, U.S.A.) at 37°C. *E. coli* strain JM109 was incubated in the LB medium at 37°C under shaking conditions at 200 rpm.

### Construction of pBSHH1-XIAP-siRNA plasmids

Two siRNAs were designed in accordance with human *XIAP* gene sequence. Oligonucleotide templates encoding XIAP siRNAs were synthesized as follows: sense XIAP1-siRNA, 5′-GATCCCCGTGGTAGTCCTGTTTCAGCTTCAAGAGAGCTGAAACAGGACTACCACTTTTTGGAAA-3′; antisense XIAP1-siRNA, 5′-AGCTTTTCCAAAAAGTGGTAGTCTGTTTCAGCTCTCTTGAAGCTGAAACAGGACTACCACGGG-3′; sense XIAP2-siRNA, 5′-GATCCCCTGGTATCCAGGGTGCANATTTCAAGAGAATTTGCACCCTGGATACATTTTTGGAAA-3′; antisense XIAP2-siRNA, 5′-AGCTTTTCCAAAAATGGTATCCAGGGTGCAAATTCTCTTGAAATTTGCACCCTGGATACCAGGG-3′. Primer sequences of XIAP1-siRNA and XIAP2-siRNA were synthesized by Shanghai Sangon Biological Engineering Technology & Services Co., Ltd. (Shanghai, China). Four synthetic sequences were separately resuspended in 10 mmol/l Tris/HCl (pH 8.0) to a final concentration of 100 µmol/l. The forward and reverse primers (a 1:1 volume mixture) were heated to 95°C for 3 min, after which these were annealed, cooled to 37°C, and preserved at –20°C. The pBSHH1 plasmid was digested with two restriction enzymes BglII and HindIII (Fermentas Thermo Fisher Scientific Inc., Waltham, MA, U.S.A.), and electrophoresed in 1% agarose. After being excised from the gel, the segments were ligated to annealing products of XIAP1-siRNA and XIAP2-siRNA, respectively. Next, competent cells of *E. coli* JM109 were transformed with ligated segments. Finally, clones were selected after identification, and they were named as pBSHH1-XIAP1-siRNA and pBSHH1-XIAP2-siRNA.

### Cell transfection

Well-cultured EC9706 and KYSE30 cells were collected by centrifugation at 1000 rpm for 5 min and resuspended in serum-free RPMI 1640 medium. pBSHH1-XIAP1-siRNA and pBSHH1-XIAP2-siRNA (4 µg each plasmid) were added into 225 µl of serum-free RPMI 1640 medium. The solution was gently mixed and maintained for 5 min, which was referred to as solution A. A total of 10 µl of Lipofectamine 2000 (Invitrogen Inc., Carlsbad, California, U.S.A.) was added into 240 µl of serum-free RPMI 1640 medium. After gentle mixing, the solution was maintained for 5 min and was named as solution B. Then solution B was slowly added and mixed with solution A. The mixed solution, named as solution C, was cultured at room temperature for 20 min. Then 500 µl of solution C was added into six-well plate, and incubated at 37°C with 5% CO_2_ for 6 h. Subsequently, the original medium was replaced with RPMI 1640 medium for another 24-h culture, followed by a selection with 400 µg/ml G418 (Amresco Inc., Solon, Ohio, U.S.A.). After 2–3 weeks, monoclonal cells were visible to naked eyes, and they were selected to conduct amplification in RPMI 1640 medium to establish stable transfected cell lines. The cells were divided into four groups: the blank control group (without any transfection), the negative control (NC) group (transfected with the empty pBSHH1 plasmid), the siRNA-enhanced group (transfected with the pBSHH1-XIAP1-siRNA plasmid), and the siRNA-decreased group (transfected with the pBSHH1-XIAP2-siRNA plasmid). After a 24-h culture, total RNA and total protein were extracted from cells in each group to detect *XIAP* mRNA and protein expressions.

The article "Down-regulation of XIAP enhances the radiosensitivity of esophageal cancer cells in vivo and in vitro" was retracted in 2021. Reasons: fabricated or falsified data; manipulated images; an official misconduct investigation; misconduct by an author.

### Reverse-transcription quantitative PCR

Total RNA was extracted from 1 × 10^5^ cells using TRIzol kit (Invitrogen Inc., Carlsbad, California, U.S.A.). The cDNA template was synthesized by reverse transcription kit (Hangzhou Bioer Technology Co., Ltd., Hangzhou, China). The reverse-transcription quantitative PCR (RT-qPCR) was performed to detect the mRNA expression of the target gene in samples. Primer sequences were as follows: XIAP, forward primer: 5′-GACAGTATGCAAGATGACGTCAAGTCA-3′ and reverse primer: 5′-GCAAAGCTTCTCCTCTTGCAG-3′; β-actin (as an internal reference gene), forward primer: 5′-CAGGGTGTGATGGTGGGTATG-3′ and reverse primer: 5′- TCCCTCTCAGCTGTGGTGG-3′. The RT-qPCR was conducted using an ABI 7500 PCR instrument (Applied Biosystems by Life Technologies., Foster City, California, U.S.A.). RT-qPCR mixture was purchased from Bio–Rad Laboratories, Inc. (Hercules, California, U.S.A.). Reaction procedures: predenaturation at 95°C for 10 min; 40 cycles of denaturation at 94°C for 30 s, annealing at 58°C for 30 s, and extension at 72°C for 1 min. The differential expression of mRNA was calculated by N = 2^−ΔΔ*C*^_t_. Here, *C*_t_ was the cycle number when the fluorescence intensity reached the settled threshold.

### Western blotting

A total of 1 × 10^5^ cells were added with 0.5 ml PBS. Then, the cells were disrupted in an ultrasonic processor (Ningbo Scientz Biotechnology Co., Ltd., Zhejiang, China). After the cells were centrifuged at 12000 rpm for 10 min, the total protein concentration in the supernatant was detected using the Bradford method. Next, the samples were adjusted to the same concentration with total protein. The same amount of supernatants was obtained and the protein was separated by 10% SDS/PAGE and transferred on to PVDF membranes at 17 V for 30 min using a Trans-Blot SD Semi-Dry Transfer Cell (Bio–Rad Inc., Hercules, California, U.S.A.). Then, the membranes were blocked with 6% (m/v) skimmed milk in PBS at room temperature for 2 h, and washed with PBST (PBS plus 0.1% (w/v) Tween-20) three times, 3 min per time. Later, the membranes were added with rabbit anti-human XIAP monoclonal antibody (Abcam Inc., Cambridge, U.K.), and incubated at room temperature for 1 h. After being washed using PBST for five times (3 min/time), the samples were incubated at room temperature for another hour with the addition of horseradish peroxidase (HRP)–conjugated goat anti-rabbit IgG (Zhongshan Golden Bridge Biotechnology Ltd., Co., Beijing, China). Finally, these samples were rinsed with PBST for five times, 3 min per time. The target proteins were visualized using HRP substrate (Bio–Rad Inc., Hercules, California, U.S.A.).

β-actin served as an internal reference, and rabbit anti-humn β-actin protein (Zhongshan Golden Bridge Biotechnology Ltd., Co., Beijing, China) as the primary antibody. The gray-scale values of XIAP and β-actin protein bands detected by Western blotting were analyzed by ImagePro Plus 6.0, and the relative expression of XIAP was expressed as the ratio of two gray-scale values (XIAP/β-actin).

The article "Down-regulation of XIAP enhances the radiosensitivity of esophageal cancer cells in vivo and in vitro" was retracted in 2021. Reasons: fabricated or falsified data; manipulated images; an official misconduct investigation; misconduct by an author.

### Radiation treatment

Cells in the logarithmic growth phase were digested with 0.25% trypsin and repeatedly disassociated to a single-cell suspension. Cells were irradiated at room temperature using a 6 MV X-ray beam from a linear accelerator (2100EX; Varian Medical Systems, Palo Alto, CA, U.S.A.), with irradiation doses of 2, 4, 6, 8, and 10 Gy, respectively, an irradiation distance of 100 cm, and an absorbed dose rate of 300 cGy/min. The cell survival and viability was determined by MTT and colony formation assay. Caspase-3 and caspase-9 activity were detected with caspase-3 activity detection kit and caspase-9 activity detection kit; and cell apoptosis was measured using flow cytometry. The experiment was repeated three times.

### MTT assay

Cells in each group were seeded into a medium containing 10 ml of fresh medium at a concentration of 5 × 10^5^ cells/ml, and incubated at 37°C in an incubator containing 5% CO_2_ for 24 h. A total of 10 µl cell counting kit-8 (CCK-8 kit; Dojindo Laboratories, Kumamoto, Japan) was added into each well, followed by 1-h culture in an incubator. Optical density (OD) at a wavelength of 490 nm (OD_490_) was detected by a microplate reader (Thermo Fisher Scientific Inc., Waltham, MA, U.S.A.). With the blank well as zero setting and EC9706 and KYSE30 cells without any transfection as control, the experiment was performed for three times. Cell survival curve was obtained with time as abscissa and OD_490_ as ordinate. Formula: cell survival rate (%) = (OD_490_ of the experiment well – OD_490_ of the blank well)/(OD_490_ of the control well – OD_490_ of the blank well) × 100%.

The article "Down-regulation of XIAP enhances the radiosensitivity of esophageal cancer cells in vivo and in vitro" was retracted in 2021. Reasons: fabricated or falsified data; manipulated images; an official misconduct investigation; misconduct by an author.

### Colony formation assay

Cells in each group were suspended, diluted, and seeded into fresh medium (10 ml) at a concentration of 50, 100, 200 cells per medium, respectively. After mixture, cells were incubated in an incubator at 37°C with 5% CO_2_ and saturated humidity for 48 h. The supernatant was discarded. Cells were washed three times by PBS, fixed in paraformaldehyde and stained with Crystal Violet for 10 min. After washing with PBS twice, staining solution was removed, and cells were dried in the air. Next, the culture dish was inverted with a transparent film (with mesh) overlaid to count the number of colonies with more than ten cells under a low-power microscope. The experiment was performed three times. The colony-forming efficiency was calculated based on the following formula: colony-forming efficiency = (the number of colony forming units/the number of inoculated cells) × 100%.

### Caspase-3 and caspase-9 activity and flow cytometry

Cells in each group were seeded into a fresh medium (10 ml) at a concentration of 5 × 10^5^ cells/ml. After being irradiated at 6 Gy and incubated at 37°C in a 5% CO_2_ incubator for 48 h, cell suspension was prepared after trypsinization, followed by centrifugation at 1000 rpm for 5 min. After washing twice with precooled PBS, cells were resuspended with 1 ml PBS and split into four tubes (0.5 ml/tube). Subsequently, 0.5 ml of caspase-3 activity assay kit and 0.5 ml of caspase-9 activity assay kit (Calbiochem, Merck KGaA, Darmstadt, Germany) was added into lysis buffer in the two tubes, respectively. The lysates were centrifuged at 12000 rpm for 5 min. A total of 100 µl supernatant was collected and reacted with 800 µl reaction buffer and 5 µl substrate Ac-DEVD-AFC at 37°C for 1 h. The fluorescence intensity was detected using a fluorospectrophotometer at a wavelength of 380 nm and emission wavelength of 430–460 nm, to calculate caspase-3 and caspase-9 activity. Cells in the other two tubes were resuspended with 500-µl binding buffer containing Annexin V-FIFC/povidone iodine (PI) apoptosis detection kit (Beyotime Biotechnology Co., Ltd., Shanghai, China). With the addition of 5 µl Annexin-FIFC, cells in this tube were incubated in the dark at 2–8°C for 15 min. Then, the cells were blended with 5 µl PI and incubated in the dark at 2–8°C for 15 min again. Cell apoptosis was determined by flow cytometry within 2 h.

The article "Down-regulation of XIAP enhances the radiosensitivity of esophageal cancer cells in vivo and in vitro" was retracted in 2021. Reasons: fabricated or falsified data; manipulated images; an official misconduct investigation; misconduct by an author.

### A nude mouse model for tumorigenesis

EC9706 cell line was selected for the establishment of a nude mouse model. Twenty male BALB/C nude mice (4-week-old) were obtained from Southern Medical University, Laboratory Animal Center. The nude mice were divided into four groups (five mice in each group) and implanted with EC9706 cells of each group (the blank control, NC, the siRNA-enhanced, and the siRNA-decreased groups), respectively. Twenty-four hours after cell transfection, cells were digested with trypsin, and washed twice using PBS. Cells were suspended in serum-free RPMI 1640 medium at a concentration of 1.5 × 10^8^ cells/ml, and injected subcutaneously into the back of the nude mouse after mixing with 0.1 ml ECM gel. Tumor was formed 7 days after implantation. Fifteen days after implantation, mice were irradiated with 6 MV X-ray at a dose of 15 Gy. After tumor formation, the tumor volume was measured once a week. Tumor volume was calculated as follows: V = π × D_long_ × D_short_^2^/6 (D_long_, long diameter; D_short_, short diameter). At the end of the sixth week, all mice were killed to measure the tumor volume and weight.

### Statistical analysis

SPSS 21.0 software (SPSS Inc., Chicago, IL, U.S.A.) was applied for data analysis. Measurement data were expressed as mean ± S.D. and a normal distribution of which was analyzed using the normality test. The comparison of measurement data was analyzed by *t*test. One-way ANOVA was used to analyze comparisons amongst multiple groups. *P*<0.05 was considered statistically significant.

## Results

### XIAP1 expressions in five EC cell lines

The results of RT-qPCR and Western blotting revealed that XIAP1 gene was overexpressed in EC9706 and KYSE30 cell lines, and down-regulated in TE10, KYSE70, and KYSE510 cell lines (Figure 1). EC9706 and KYSE30 cell lines were selected for further experiments.

**Figure 1:** RT-qPCR and Western blotting results of XIAP1 expressions of EC9706, TE10, KYSE70, KYSE510, and KYSE30 cell lines (**A**) RT-qPCR results of the *XIAP1* mRNA expressions in different cell lines; (**B**) Western blotting results of thee XIAP1 protein expressions in different cell lines; (**C**) protein bands of XIAP1 and β-actin gene of different cell lines by Western blotting.

### Establishment and identification of pBSHH1-XIAP-siRNA plasmids

The annealing products of XIAP1-siRNA and XIAP2-siRNA DNA templates (Figure 2A) were connected with the segments in the pBSHH1 vector, and transformed into *E. coli* JM109 competent cells. The positive transformants and plasmids were extracted and then identified using enzymes BglII and HindIII (Figure 2B). The results revealed that XIAP1 siRNA and XIAP2 siRNA DNAs were successfully connected with the pBSHH1 and that the recombinant plasmids were named as pBSHH1-XIAP1-siRNA and pBSHH1-XIAP2-siRNA. Sequencing of two recombinant plasmids was conducted by Shanghai Sangon Biological Engineering Technology & Services Co., Ltd. (Shanghai, China). The results suggested the hairpin structure and designed sequences of siXIAP1 and siXIAP2 were totally identical.

The article "Down-regulation of XIAP enhances the radiosensitivity of esophageal cancer cells in vivo and in vitro" was retracted in 2021. Reasons: fabricated or falsified data; manipulated images; an official misconduct investigation; misconduct by an author.

**Figure 2:** Establishment and identification of pBSHH1-XIAP-siRNA plasmids (**A**) Electrophoresis images of the annealing products of siRNA single-stranded oligonucleotide templates. M: molecular weight maker; (1) the annealing products of single-stranded oligonucleotide XIAP1; (2) the annealing products of single-stranded oligonucleotide XIAP2. (**B**) The identification of pBSHH1-XIAP-siRNA and pBSHH1-XIAP2-siRNA plasmids by enzyme digestion; M, molecular weight maker; (1) pBSHHI-XIAP1-siRNA; (2) pBSHH1-XIAP2-siRNA.

### *XIAP* mRNA and protein expressions of EC9706 and KYSE30 cell lines in the four groups

The mRNA and protein expressions of XIAP amongst the four groups were detected using RT-qPCR and Western blotting. The results showed that the mRNA and protein expressions of XIAP in the NC group were not significantly different from these in the blank control group (all *P*>0.05). Compared with the NC group, *XIAP* mRNA and protein expressions in the siRNA-enhanced and siRNA-decreased groups were decreased (all *P*<0.05). Moreover, expressions of *XIAP* mRNA and protein in the siRNA-enhanced group were lower than those in the siRNA-decreased group (all *P*<0.05, Figure 3).

**Figure 3:** *XIAP* mRNA and protein expressions of EC9706 and KYSE30 cell lines in the four groups (**A**) *XIAP* mRNA expressions of EC9706 cell line in the four groups; (**B**) band analysis of XIAP protein of EC9706 cell line in the four groups analyzed by Western blotting; (**C**) XIAP protein expressions of EC9706 cell line in the four groups; (**D**) *XIAP* mRNA expressions of KYSE30 cell lines in the four groups; (**E**) band analysis of XIAP protein of KYSE30 cell line in the four groups analyzed by Western blotting; (**F**) XIAP protein expressions of KYSE30 cell line in the four groups; *, *P*<0.05 compared with the NC group; ^#^, *P*<0.05 compared with the siRNA-enhanced group.

### Radiosensitivity of EC cells of EC9706 and KYSE30 cell lines in the four groups

The radiosensitivity was detected after X-ray radiation. The MTT results in Figure 4 showed that with increasing dose, cell survival rates were decreased in all four groups (all *P*<0.05). The cell survival rate showed no significant difference between the NC group and the blank control group (all *P*>0.05). Compared with the NC group, cell survival rates were decreased significantly in the siRNA-enhanced and siRNA-decreased groups (all *P*<0.05). Besides, the cell survival rate in the siRNA-enhanced group was lower than that in the siRNA-decreased group (both *P*<0.05). The colony formation assay suggested that colony-forming efficiency was not significantly different between the NC group and the blank control group (both *P*>0.05). When compared with the NC group, there was a decrease in colony-forming efficiency in the siRNA-enhanced group (both *P*<0.05). Furthermore, the siRNA-decreased group exhibited an increase in colony-forming efficiency when compared with the siRNA-enhanced group (both *P*<0.05).

The article "Down-regulation of XIAP enhances the radiosensitivity of esophageal cancer cells in vivo and in vitro" was retracted in 2021. Reasons: fabricated or falsified data; manipulated images; an official misconduct investigation; misconduct by an author.

**Figure 4:** Radiosensitivity of EC9706 and KYSE30 cell lines in the four groups (**A**) The curve of cell survival rate of EC9706 cell line in the four groups detected by MTT assay; (**B**) the colony-forming efficiency of EC9706 cell line in the four groups assessed by colony formation assay; (**C**) the curve of cell survival rate of KYSE30 cell line in the four groups detected by MTT assay; (**D**) the colony-forming efficiency of KYSE30 cell line in the four groups assessed by colony formation assay; *, *P*<0.05 compared with the NC group; ^#^, *P*<0.05 compared with the siRNA-enhanced group.

### Caspase-3 and caspase-9 activity and apoptosis rate of EC9706 and KYSE30 cell lines in the four groups

Caspase-3 and caspase-9 activity detection results showed no significant difference between the NC and blank control groups (all *P*>0.05). Caspase-3 and caspase-9 activity in the siRNA-enhanced and siRNA-decreased groups were elevated in comparison with the NC group (all *P*<0.05). Furthermore, the siRNA-enhanced group exhibited higher caspase-3 and caspase-9 activity than the siRNA-decreased group (all *P*<0.05, Figure 5).

**Figure 5:** Caspase-3 and caspase-9 activity of EC9706 and KYSE30 cell lines in the four groups (**A**) Caspase-3 activity of EC9706 cell line in the four groups; (**B**) caspase-9 activity of EC9706 cell line in the four groups; (**C**) caspase-3 activity of KYSE30 cell line in the four groups; (**D**) caspase-9 activity of KYSE30 cell line in the four groups; *, *P*<0.05 compared with the NC group; ^#^, *P*<0.05 compared with the siRNA-enhanced group.

The results of cells’ apoptosis in Figure 6 suggested that cell apoptotic rate in the NC group was not significantly different from that in the blank control group (both *P*>0.05). The apoptotic rates in the siRNA-enhanced and siRNA-decreased groups were higher than those in the NC group (all *P*<0.05). And the apoptotic rate in the siRNA-enhanced group was evidently higher than that in the siRNA-decreased group (both *P*<0.05).

The article "Down-regulation of XIAP enhances the radiosensitivity of esophageal cancer cells in vivo and in vitro" was retracted in 2021. Reasons: fabricated or falsified data; manipulated images; an official misconduct investigation; misconduct by an author.

**Figure 6:** Apoptotic rates of EC9706 and KYSE30 cell lines in the four groups (**A**) Apoptotic cells of EC9706 cell line in the four groups determined by flow cytometry; (**B**) apoptosis rate of EC9706 cells in the four groups; (**C**) apoptotic cells of KYSE30 cell line in the four groups determined by flow cytometry; (**D**) comparison of apoptosis rate of KYSE30 cells in the four groups; *, *P*<0.05 compared with the NC group; ^#^, *P*<0.05 compared with the siRNA-enhanced group.

### Tumor volume and weight of nude mice of EC9706 cell line in the four groups after EC cell implantation

The tumor growth in nude mice in each group was presented in Figure 7. The results revealed that the transplanted tumor could be observed 1 week after EC cell implantation. As time progressed, the tumor volume in the NC group showed no significant difference from that in the blank control group (*P*>0.05), while the tumor volumes in the siRNA-enhanced and siRNA-decreased groups were decreased compared with the NC group (both *P*<0.05). Six weeks after EC cell implantation, the mice were killed to measure the tumor weight. It was shown that the tumor weights of mice in the blank control, NC, siRNA-enhanced, and siRNA-decreased groups were 2.07, 1.89, 0.68, and 1.33 g, respectively. The NC group presented greatly increased tumor weight than both the siRNA-enhanced and siRNA-decreased groups (both *P*<0.05), and the tumor weight in the siRNA-enhanced group was decreased in the siRNA-decreased group (*P*<0.05), indicating that down-regulation of XIAP expression might inhibit tumor growth. Moreover, the lower the XIAP expression was, the more effective it was to suppress tumor growth.

**Figure 7:** Tumor volume and weight of nude mice of EC9706 cell line in the four groups after EC cell implantation (**A**) Growth curves of tumor volume of nude mice in the four groups after EC cell implantation; (**B**) tumor weight of nude mice in the four groups after EC cell implantation. *, *P*<0.05 compared with the NC group; ^#^, *P*<0.05 compared with the siRNA-enhanced group. (**C**) Transplanted tumors in the four groups.

## Discussion

XIAP is often reported to be closely correlated with undesirable clinical outcomes in anticancer therapies with a high expression in malignant cells [20,21]. Malignant cells with overexpressed XIAP have been found to be highly resistant to standard radiotherapy and chemotherapy [22]. Since radiation resistance reduced the therapeutic efficacy when treating EC patients, and thus, it is necessary to conduct more studies to develop a new strategy to enhance the radiation sensitivity of antineoplastic therapies and elevate survival rate of EC patients [23]. Consistently, the present study revealed that siRNA-mediated *XIAP* gene silencing could boost the radiosensitivity of EC cell line.

The article "Down-regulation of XIAP enhances the radiosensitivity of esophageal cancer cells in vivo and in vitro" was retracted in 2021. Reasons: fabricated or falsified data; manipulated images; an official misconduct investigation; misconduct by an author.

The mRNA and protein expressions of XIAP were detected by RT-qPCR and Western blotting in EC9706 and KYSE30 cells. The results demonstrated that no matter what in the siRNA-enhanced group or in the siRNA-decreased group, *XIAP* mRNA and protein expressions were evidently decreased when compared with the NC group; especially, the siRNA-enhanced group exhibited even lower expressions of *XIAP* mRNA and protein than the siRNA-decreased group. Previously, Obexer et al. [24] has reported that XIAP is highly expressed in most malignant tumor cells and expressions of *XIAP* mRNA and protein are closely associated with the sensitivity to cancer therapies and overall survival. Additionally, caspase-3 and caspase-9 activity and cell apoptosis were increased in the siRNA-enhanced and siRNA-decreased groups after radiation treatment. Caspases are pivotal enzymes for cell apoptosis that are conducted via the caspases-mediated cascade amplification reactions, and wherein caspase-3 and caspase-9 are the key initiators of cell apoptotic process [25,26]. XIAP binding to caspases suppresses the proteolytic degradation which represents the final enforcement of apoptosis, and the knockdown of XIAP expression targetted and silenced by siRNA enhances the apoptosis and sensitivity in tumor cells [27], suggesting that siRNA targetting XIAP could reinforce cell apoptosis and radiation sensitivity of EC cells to radiotherapy with efficient down-regulation of XIAP expression [28]. In the present study, these findings also proved that *XIAP* gene silencing functioned in tumor cells by binding to caspase-3, thereby enhancing cell apoptosis.

In addition, results of MTT assay and clone formation assay indicated that both cell survival rate and colony forming efficiency were indeed suppressed after radiotherapy when XIAP was blinded by siRNA. Knockdown of the vital gene related to EC via siRNA can guarantee better efficacy of EC patients in radiotherapy by improving the radiation sensitivity of tumors [23]. The overexpressed XIAP results in poor clinical response, but decreased XIAP expressions are associated with better prognosis [29]. XIAP has been characterized, as a concentration-dependent responder to apoptotic and bioenergetic stresses, upstream of caspase activation [30]. XIAP dysregulation in papillary thyroid carcinoma is also reported to confer an aggressive phenotype with poor outcome [31]. Similarly, a study demonstrates that reduction in XIAP expression can sensitize malignant tumor cells to antineoplastic therapies in EC via binding to caspases and enhancing apoptosis [28]. Furthermore, rectal cancer cells which survive in therapies are resistant to radiochemotherapy by elevating the protein levels of XIAP [32]. In consistent with our findings, Zhang et al. [33] also show that the inhibition of XIAP can reinforce radiation sensitivity and heighten therapeutic outcome of EC treatment, wherein EC cells transfected with XIAP-siRNA presents lower XIAP expressions by activating caspase-3 to increase apoptosis, so it could sensitize cancer cells to chemotherapeutics contributing to a better clinical response. Here, the study also indicated that an enhancement in the sensitivity to radiotherapy would be achieved by *XIAP* gene silencing. Potent siRNA can cause effective reduction in both mRNA and protein expressions of XIAP, and it is one promising option to weaken the resistance of cancer cells to antineoplastic agents [34]. In the present study, a nude mice model of EC *in vivo* was conducted to detect the radiosensitivity with the siRNA knockdown of XIAP by examining the volume and weight of transplanted tumors. Compared with the NC group, decreased volume and weight of transplanted tumors were found in mice after radiation therapy with siRNA targetting XIAP.

The article "Down-regulation of XIAP enhances the radiosensitivity of esophageal cancer cells in vivo and in vitro" was retracted in 2021. Reasons: fabricated or falsified data; manipulated images; an official misconduct investigation; misconduct by an author.

To conclude, mRNA and protein expressions of XIAP were decreased via siRNA targetting, which leads to increases in cell survival rate and colony formation efficiency with increases in cell apoptosis and caspase-3 and caspase-9 activity. It also contributed to the reduced tumor size and tumor weight. Therefore, XIAP expression might be an effective diagnostic factor, and *XIAP* gene may functions as a novel genetic target for the treatment of EC patients via siRNA so as to enhance the radiosensitivity of EC cells. Meanwhile, more investigations are required due to the limitations of other factors failed to mention in our study which affect the overall radiosensitivity in EC patients.

## Abbreviations

EC: esophageal cancer
FITC: fluorescein isothiocyanate
HRP: horseradish peroxidase
IAP: inhibitor of apoptosis protein
NC: negative control
OD_490_: optical density at a wavelength of 490 nm
PBST: PBS plus 0.1% (w/v) Tween-20
PI: povidone iodine
RPMI 1640: Roswell Park Memorial Institute 1640
RT-qPCR: reverse-transcription quantitative PCR
XIAP: X-chromosome-linked inhibitor of apoptosis
